# CYR61, a potential biomarker of tumor inflammatory response in epithelial ovarian cancer microenvironment of tumor progress

**DOI:** 10.1186/s12885-019-6321-x

**Published:** 2019-11-25

**Authors:** Jun Shi, Rongfen Huo, Ningli Li, Haichuan Li, Tianhang Zhai, Huidan Li, Baihua Shen, Jing Ye, Ruojin Fu, Wen Di

**Affiliations:** 1 Department of Obstetrics and Gynecology, Renji Hospital, School of Medicine, Shanghai Jiaotong University, Shanghai, 200127 China; 2 Shanghai Key Laboratory of Gynecologic Oncology, Shanghai, 200127 People’s Republic of China; 3 Shanghai Institute of Immunology, School of Medicine, Shanghai Jiao Tong University, Shanghai, 200025 China

**Keywords:** Epithelial ovarian cancer, Cyr61, Tumor-associated inflammatory microenvironment, Tumor progression

## Abstract

**Background:**

Recent studies have found that inflammatory response is involved in the pathogenesis of ovarian cancer. Advanced ovarian cancer is often presented with ascites that is rich in cytokines, inflammatory factors or cancer cells. Therefore, it is important to study the microenvironment of ascites in order to further clarify the occurrence and progression of ovarian cancer. As a pro-inflammatory factor, the Cyr61 expression patterns are inconsistent in human tumors. Although it has been reported that Cyr61 is related to the progression of ovarian cancer, its specific mechanism is not yet clear. This study sought to evaluate the Cyr61 levels of ascites, serum and different tissues of ovarian cancer to explore the potential association of Cyr61with the tumor-associated inflammatory microenvironment of EOC.

**Methods:**

Tumor specimens were procured from patients with ovarian serous cystadenocarcinoma and ovarian serous cystadenoma. Cyr61 and IL-6 levels of serum or ascites were determined by ELISA (Enzyme-Linked ImmunoSorbent Assay), while Cyr61 expressions of different ovarian tumor tissues were evaluated by IHC (Immunohistochemistry). Then the correlation of Cyr61 level in ascites with clinicopathologic features was analyzed. And other laboratory data were obtained from medical records.

**Results:**

Both in ascites and serum, significantly higher Cyr61 levels were found in ovarian serous cystadenocarcinoma. In malignant ascites, higher Cyr61 level of ovarian serous cystadenocarcinoma was more closely associated with FIGO stage, initial tumor size > 10 cm and the residual tumor size. And the increased IL-6 level was linearly related to Cyr61 level. Moreover, the serum levels of Cyr61, IL-6 and CRP in advanced stage of ovarian cancer were much higher than those in early stage. Lastly, the IHC data demonstrate that Cyr61 expression of ovarian serous adenocarcinoma was higher than that of ovarian serous cystadenoma, but it was lower than the paired metastatic lesions.

**Conclusions:**

As a pro-inflammatory factor, increased ascites Cyr61 level is associated with FIGO stage, initial tumor size > 10 cm and the residual tumor size. Moreover, serum Cyr61 may be used as a potential marker for EOC inflammatory response. Finally, Cyr61 may be involved in the process of tumor metastasis and progression by producing IL-6 and CRP in the EOC inflammatory microenvironment.

## Background

Epithelial ovarian cancer (EOC) is the most lethal gynecological cancer [1]. Due to its unclear pathogenesis and lack of early detection method, about 75% of EOC patients have advanced-stage at initial diagnosis, and the effect of treatment and prognosis are both not good. Therefore, further exploration of the mechanism of EOC onset and later peritoneal metastasis is of great significance for finding new earlier diagnostic biomarkers and new target of blocking tumor metastasis.

In modern tumor biology, it is well known that tumor microenvironment is a key factor in malignant tumor development and metastasis. Moreover, studies have shown that the tumor-associated inflammatory microenvironment constructed by a variety of inflammatory factors secreted by tumors and stromal cells (such as fibroblasts), regulates the growth, invasion and metastasis of tumor cells, and ultimately directly determine the malignant properties of tumor cells [2–6]. It is reported that the inflammatory response involved in the pathogenesis of ovarian cancer, for the malignant ascites containing a large number of exfoliated cancerous cells, which may become a source of cancer cells metastasis and peritoneal implantation [7–9]; high concentrations of pro-inflammatory cytokines such as IL-6, IL-8 contained in ascites can promote cancer cell growth and metastasis, which all can accelerate the progress of the disease, reducing the treatment effect and worsening the prognosis [10–12]. However, with further research, some other factors should be found to be more decisive in the formation and maintain of inflammatory microenvironment, and might play very important role in tumor growth by promoting secretion of some inflammatory cytokines.

Cyr61 (cysteine-rich protein 61) is the first identified member of the CCN family, also known as CCN1. It is a 40 kDa secreted matrix protein and is known to play an important role in cell proliferation, adhesion, inducing angiogenesis and other important physiological activities [13–16]. Moreover, Cyr61 has been reported recently to participate in tumor development, promoting vascular proliferation or increasing tumor cell proliferation and migration [17–19]. What’s more, Cyr61 may mainly promote secretion of IL-6, IL-8, pro-IL-1β et al. to enhancing inflammation and tissue damage as a novel pro-inflammatory cytokine [20–24]. In human tumor inflammatory microenvironment, IL-6 has also been proved to stimulate the migration and invasion of cancer cells of breast cancer, pancreatic cancer and osteosarcoma [25–27]. Similarly, some studies about ovarian cancer have found that IL-6 also promotes the development of tumor, which is closely related to the prognosis [28, 29]. So Cyr61 may be a protagonist in tumor inflammatory microenvironment.

For ovaries, there is a dynamic inflammatory reaction in each ovulation cycle. And recent studies have shown that the incidence of ovarian cancer is closely related to the wound repair caused by continuous ovulation. So it is of great significance to explore the inflammatory response involved in the formation and maintain of ovarian cancer microenvironment for the early diagnosis and appropriate treatment. Nevertheless, whether Cyr61 plays a pivotal role in the inflammation microenvironment processes of ovarian carcinoma development has not been explored yet. In this study, the Cyr61 expression patterns in serum, ascites and tissue of EOC were evaluated. At the same time, the correlation of Cyr61 with IL-6, other inflammatory markers and clinicopathologic features was analyzed respectively to explore the potential association of Cyr61with EOC progression in the tumor-associated inflammatory response.

## Methods

### Patient samples

Between January 2014 and December 2016, tumor tissue, ascites (or peritoneal lavage fluid) and peripheral blood samples were obtained from 66 patients with ovarian serous cystadenocarcinoma (mean age: 58.24 ± 0.99 years) and 18 patients with ovarian serous cystadenoma (mean age: 43.06 ± 2.16 years) of the Department of and Obstetrics and Gynecology, Renji Hospital, School of Medicine, Shanghai Jiao Tong University, Shanghai, China.

Two experienced pathologists reviewed the paraffin pathology respectively. Stage is based on the 2014 International Federation of Gynecology and Obstetrics (FIGO) criteria. The exclusion criteria were inadequate follow-up data, chemotherapy before operation and combined with inflammatory or immune disease. Ascites fluid was obtained at the time of initial surgery and centrifuged at 1000 g for 15 min. The peripheral blood samples were taken on the morning before the operation. Ascites supernatants and all serum samples were stored at − 80 °C until assayed. Tissue specimens were snap-frozen in liquid nitrogen.

This study was approved by ethics committee of Renji Hospital, School of Medicine, Shanghai Jiao Tong University and it was in compliance with the Helsinki Declaration. All the patients gave written informed consent for participation in the study.

### Enzyme linked Immunosorbent assay (ELISA)

ELISA kit (Cyr61, Cat Log#: DY4055; IL-6, Cat Log#: HS600B; R&D System, MN, USA) for quantitatively detecting serum and ascites of Cyr61, IL-6 were used according to the manufacturer’s instructions. Briefly, the samples were added in duplicate to the wells of the microtiter plate coated with an antibody against Cyr61 or IL-6 with horseradish peroxidase-conjugate. Then, absorbance at the 450 nm in each microwell was measured using spectrophotometer. Each cytokine analysis was simultaneously performed on all patients and control serum, thereby avoiding a possible defrosting/refreezing bias.

### Laboratory analyses

Laboratory data were obtained from medical records; Blood samples were originally taken using standard procedures and analyzed in the course of routine treatment. Blood routine examination was quantified by Sysmex kit. C-reactive protein (CRP) was quantified by Aristo (AR51200) kit.

### Immunohistochemical (IHC) stain and data analysis

Ovarian serous cystadenoma and serous cystadenocarcinoma tissues were fixed in 4% paraformaldehyde, embedded in paraffin and sectioned. The Cyr61 expression was determined by immunohistochemistry assay. Briefly, the tissue samples were stained with mouse anti-human Cyr61 mAb at a concentration of 1:200 followed by HRP conjugated goat anti-mouse secondary antibody according to previous reports [30, 31]. Cyr61 expression evaluated by two independent observers though examining the Cyr61-stained tissue, and a consensus score was determined for each specimen.

A positive reaction was scored into 4 grades, according to the intensity of the staining: 0, +, ++, and +++. The percentages of Cyr61-positive cells were also scored into 5 categories: 0 (≤5%), 1 (6–25%), 2 (26–50%), 3 (51–75%) and 4 (76–100%). The final score, calculated as the product of the intensity score multiplied by the percentage score, was classified as follows: 0 for negative; 1–3 for weak; 4–7 for moderate; and 8–12 for strong.

### Statistical analysis

Data were presented as mean ± SD or n (%), differences between groups were analyzed by unpaired Student’s t test. Comparisons of categorical variables were conducted using x^2^ testing. For all statistical analyses, 2-tailed *P* < 0.05 was considered statistically significant. All statistical analyses were performed using the Statistical Package for the Social Sciences, version 13.0 (SPSS Inc., Chicago, IL, USA) or GraphPad Prism 4.0 (GraphPad Software, San Diego, CA).

## Results

### Higher Cyr61 level was found in ascites than in serum of ovarian serous cystadenocarcinoma

Both in ascites and serum, significantly higher Cyr61 levels were found in the malignant ovarian tumor (Fig. 1).

**Fig. 1:** Expression levels of Cyr61 in ascites and serum of ovarian benign and malignant tumor *Cyr61 levels in ascites and serum of ovarian serous adenocarcinoma patients (n = 66) were significantly higher than those of ovarian serous cystadenoma patients (n = 18). And the ascites Cyr61 level was much higher than that of serum*

In ascites, the Cyr61 level of ovarian serous cystadenocarcinoma (*n* = 66) and serous cystadenoma (*n* = 18) was 1624.33 ± 191.92 cf. 230.11 ± 25.63 pg/ml respectively (*p* < 0.001); in serum, the Cyr61 level was 77.21 ± 4.81 cf. 13.32 ± 3.14 pg/ml, correspondingly (*p* < 0.001).

Moreover, the same patient with ovarian serous cystadenocarcinoma, ascites of Cyr61 level was much higher than its serum level.

### High ascites Cyr61 level associated with clinicopathologic features of ovarian serous cystadenocarcinoma

Tumor ascites microenvironment may reflect the tumor characteristics and its progress. So ascites Cyr61 was analyzed to clear its relationships with the clinicopathologic features of ovarian serous cystadenocarcinoma. Multiple regression analysis showed that.

Ascites Cyr61 level was more closely associated with FIGO stage (*p* = 0.001), initial tumor size > 10 cm (*p* = 0.002) and the residual tumor size (*p* = 0.025). But there was no correlation with the tumor histological grade (*p* = 0.539), total ascites volume (*p* = 0.124), ascites contains tumor cells (*p* = 0.124), vascular invasion (*p* = 1.756) and lymph node metastasis (*p* = 1.475) (Table 1).

**Table 1:** Correlation of the clinicopathologic features and ascites Cyr61 level of ovarian serous adenocarcinoma

Clinicopathologic factors	Categorization	Number (%)	Cyr61 (pg/ml)	*P* value
FIGO stage	I-II	14 (21.1)	698.74 ± 87.12	0.001
	III-IV	52 (78.9)	2054.23 ± 132.09^*^	
Initial tumor size (cm)	< 10	45 (68.2)	910.81 ± 98.31	0.002
	≥10	21 (31.8)	2125.66 ± 154.38^*^	
Ascites volume (ml)	< 500	9 (13.6)	1416.41 ± 102.37	0.124
	≥500	57 (86.4)	1760.65 ± 154.64	
Residual tumor (cm)	< 1	54 (81.8)	1031.64 ± 78.31	0.025
	≥1	12 (18.2)	2097.30 ± 174.69^*^	
Lymphatic invasion	–	60 (90.9)	1936.22 ± 191.37	1.475
	+	6 (9.1)	2128.37 ± 478.26	
Vascular invasion	–	62 (93.9)	2117.11 ± 201.39	1.756
	+	4 (6.1)	2403.74 ± 345.21	
Ascites tumor cells	–	57 (86.4)	1613.62 ± 119.27	0.124
	+	9 (13.6)	1736.28 ± 114.30	

### High ascites IL-6 level is associated with Cyr61 in the inflammatory microenvironment of ovarian serous cystadenocarcinoma

As a new pro-inflammatory factor, Cyr61 can regulate the expression of cytokines in inflammatory environment and it was correlated with tumor stage. So the ascites Cyr61 and IL-6 levels of ovarian serous cystadenocarcinoma were detected, respectively.

Ascites Cyr61 and IL-6 levels of advanced stage were (2199.86 ± 116.24 pg/ml, 3227.42 ± 147.82 pg/ml) both higher than those of early stage (778.98 ± 47.25 pg/ml, 1422.32 ± 74.69 pg/ml) (Fig. 2A).

**Fig. 2:** Cyr61 and IL-6 levels in ascites of different (the early or advanced) stage of ovarian cancer patient and the correlation. *In the patient with ovarian serous adenocarcinoma, ascites Cyr61 and IL-6 levels of the advanced stage (n = 52) were both higher than those of the early stage (n = 14). And the increased IL-6 expression was linearly related to Cyr61 level in malignant ascites*

And the increase of IL-6 level in ascites was linearly related to Cyr61 level (Fig. 2B).

### Expressions of serum Cyr61 and inflammatory markers in different stages of ovarian cancer

Inflammation is a reaction in the process of tumor development. We further examined the expression patterns of Cyr61, IL-6, CRP and neutrophil percentage in peripheral blood of patient with early or advanced stage of ovarian serous cystadenocarcinoma.

In addition to Cyr61 and IL-6, CRP serum level in advanced ovarian cancer was significantly higher than those in the early stage. However, the proportion of neutrophils of the advanced stage patients was a little higher than that in early stage, but there was no statistical difference (Table 2).

**Table 2:** Inflammatory markers in peripheral blood of ovarian cancer patient with different stages

Stage	Cyr61 (pg/ml)	IL-6 (pg/ml)	CRP (mg/L)	Neutrophils (%)
Early stage	52.55 ± 13.93	67.23 ± 17.43	7.77 ± 1.10	67.45 ± 2.37
Advanced stage	120.76 ± 22.35	212.47 ± 40.27	23.18 ± 4.48	73.56 ± 2.21
P value	0.031	0.015	0.004	1.247

### Cyr61 expression patterns in ovarian serous tumor

18 cases of ovarian serous cystadenoma, 66 cases of ovarian serous adenocarcinoma and 20 cases of its paired metastatic lesions were evaluated using IHC to confirm Cyr61expression patterns in ovarian caner (Fig. 3 and Table 3).

**Fig. 3:** Cyr61 expression patterns in the different tissues of ovarian tumor by immunohistochemistry. **a** *Benign ovarian cyst* (*ovarian serous cystadenoma) showed weak Cyr61 expression.* **b** *High grade of ovarian serous adenocarcinoma showed moderate degree Cyr61 expression.* **c** and **d** *High grade of ovarian serous adenocarcinoma of the same patient of primary and paired metastatic site showed the moderate and strong degree Cyr61 expression, respectively*

**Table 3:** Correlation of the pathological features and Cyr61 expression positive rate

Pathological type		Cyr61 expression				
		Negative (0)	Weak (1–3)	Moderate (4–7)	Strong (8–12)	Positive rate
Ovarian serous cystadenoma (n = 18)		9	8	1	0	5.56
Ovarian serous adenocarcinoma (n = 66)	G1/G2 (*n* = 7)	0	3	4	0	57.14**
	G3 (*n* = 59)	0	6	38	15	89.83**
Paired Metastatic site (*n* = 20)		0	0	1	19	95.00*

Positive rate: including moderate and strong of the intensity score (≥4)

**: Ovarian serous cystadenoma cf. Ovarian serous adenocarcinoma (*p* < 0.01);

*: Paired Metastatic site cf. Ovarian serous adenocarcinoma (*p* < 0.05)

Cyr61 expression positive rate (≥4 scores) of ovarian serous cystadenoma was significantly lower than the ovarian cancer (*p* < 0.01). Further, the positive rate of its paired metastatic lesions of was higher than the primary adenocarcinoma (*p* < 0.05).

## Discussion

The latest research results showed that there were six characteristics of the pre-metastasis microenvironment including immunosuppression, inflammatory response, enhanced angiogenesis and permeability, lymphangiogenesis, organotropy and reprogramming. It indeed indicated that the inflammatory reaction was an indispensable part of tumor progress [32]. Further, recent studies have confirmed that inflammatory microenvironment is an essential environment for tumor cells survive. In the inflammatory microenvironment, different extracellular matrix, inflammatory factors and stromal cells interact with tumor cells to promote tumor proliferation and metastasis [33–37]. The malignant ascites of ovarian cancer is a huge tumor microenvironment with its complex composition, which can enhance the ability of tumor to deteriorate [38–40].

Since previous studies have shown that the incidence of ovarian cancer is closely related to periodic ovulation and the continuous repair of ovarian surface tissues damage, it was found that the inflammatory microenvironment had a direct regulatory effect on ovarian cancer development. For various inflammatory reactions are accompanied with the process of the ovulation, all sorts of secreted cytokines and chemokine may form the microenvironment together, and it can promote the activation of oncogenes and cell carcinogenesis. So it can reveal the early events of ovarian cancer and the biological characteristics of the tumor cells. On the other hand, to be an ovarian cancer cell, it is also affected daily by physiological cycle and corresponding inflammatory changes, accelerating tumor progression. Therefore, the inflammatory microenvironment is essential for ovarian cancer [41–44].

As a novel pro-inflammatory factor, Cyr61 has been found to paly a key promoter to maintain the inflammatory microenvironment in some inflammatory and autoimmune diseases. Recently, it is interesting that “interstitium” is found to be one of the largest human organs. It is linked together to form a network supported by a strong, flexible protein network, filled with fluids in the human body. As a “highway”, full of the flowing fluids in the body, “interstitum” may help cancer cells metastasis [45]. Therefore, as one of the important interstitial proteins, Cyr61might act as a mediator in the inflammatory microenvironment of tumor. In order to analyze the role of Cyr61 play in the inflammatory microenvironment of ovarian cancer, we detected the Cyr61 level in ascites and serum of patients with ovarian serous adenocarcinoma. The Cyr61 level not only in ascites but also in serum of ovarian serous adenocarcinoma was higher than that of ovarian serous cystadenoma.

What’s more, about ovarian serous adenocarcinoma, Cyr61 level of ascites was higher than that of serum, which fully demonstrated that Cyr61 might be one of the important components in malignant ascites. And multiple regression analysis showed that Cyr61 level in ascites of ovarian serous adenocarcinoma only related to the initial tumor size, FIGO stage and surgical residual tumor size, which indicates that the increased Cyr61 level closely associated with tumor proliferation and metastasis. Further, IHC was used to analyze the expression of Cyr61 in ovarian serous adenocarcinoma tissues at different stages of progression. The results showed that the Cyr61 expression of metastatic tumor lesions (peritoneal foci) was higher than that of the primary lesions, which may signify Cyr61 playing a vital role in peritoneal metastasis.

As it is well known that IL-6 acts as promoter of tumor development and metastasis by composing inflammatory environment [46, 47]. To be the up-stream factor, Cyr61 was reported that it really promoted IL-6 secretion in the microenvironment of some inflammatory and autoimmune diseases. To explore the hypothesis that Cyr61 might also promote IL-6 production by tumor cells, then together with other factors, forming a tumor-associated inflammatory microenvironment to promote tumorigenesis, we examined the IL-6 level of ascites in ovarian serous adenocarcinoma patients and analyzed its correlation with Cyr61. The results showed that the levels of Cyr61 and IL-6 in advanced stage were significantly higher than those in early stage, which indicated that the later of the disease, the higher of Cyr61 and IL-6 levels. Further analysis showed that elevated level of IL-6 was positively correlated with elevated Cyr61 level, suggesting a synergistic effect between them in the development of tumor inflammation microenvironment.

Latest research suggested that there must be a series of special inflammatory response during the initial stage of the human tumor. Clinically, there are some commonly used biomarkers in the body’s inflammatory response, for example, white blood cells, neutrophils, CRP [48] and so on. Among them, neutrophils are the earliest to reach the site of inflammatory response [49]. It is very interesting that Cyr61 (early event) could recruit neutrophils to target sites by up-regulation IL-8 production by tissue cells at the site of inflammation. However, whether Cyr61 can mediate cytokines production and neutrophil infiltration in tumor tissues cells has not been reported yet. So we analyzed the changes of Cyr61, CRP and the percentage neutrophils in the peripheral blood of ovarian tumor. In addition to Cyr61 and IL-6, CRP serum level in advanced ovarian serous adenocarcinoma was significantly higher than those in early stage, but there was no correlation with Cyr61level. And the increasing trend of the proportion neutrophils was consistent with that of Cyr61 level. The higher level of Cyr61was, the higher percentage neutrophils became. Thus it can be seen that Cyr61may mediate neutrophil infiltration and CRP product in advanced ovarian serous adenocarcinoma just like it acts in the inflammation or autoimmune diseases. However, the specific signaling pathway remains to be studied in the near future.

## Conclusion

Our study has systematically analyzed the important role of Cyr61 as a tumor related inflammatory factor in promoting the development of ovarian cancer microenvironment.

As a pro-inflammatory matrix protein, Cyr61 expression is increasing in ovarian serous adenocarcinoma, increasing in the advanced stage, and increasing in its metastatic tumor, which suggested that Cyr61 is closely associated with the development and metastasis of EOC. More importantly, Cyr61 may paly regulation action in the upstream for tumor inflammatory microenvironment formation and maintain, especially for IL-6 expression. And as a new tumor associated inflammatory marker, Cyr61 might be a potential target and biomarker in the diagnosis, treatment and prediction of EOC, but it needs to be further study.

## Data Availability

The data was collected and saved in hospital’s medical history management center. Due to the legitimate protection of patients’ privacy, our information is not available on public or any private websites, but is available from the corresponding author on reasonable request.

## Abbreviations

EOC: Epithelial ovarian cancer
FIGO: Federation of Gynecology and Obstetrics
ELISA: Enzyme Linked Immunosorbent Assay
CRP: C-reactive protein

## References

[1] Siegel RL, Miller KD, Jemal A (2018). Cancer statistics, 2018. CA Cancer J Clin.

[2] Coussens LM, Werb Z (2002). Inflammation and cancer. Nature..

[3] Kulbe H, Thompson R, Wilson JL, Robinson S, Hagemann T, Fatah R (2007). The inflammatory cytokine tumor necrosis factor- α generates an autocrine tumor-promoting network in epithelial ovarian cancer cells. Cancer Res.

[4] Joyce Johanna A., Pollard Jeffrey W. (2008). Microenvironmental regulation of metastasis. Nature Reviews Cancer.

[5] Kulbe H, Chakravarty P, Leinster DA, Charles KA, Kwong J, Thompson RG (2012). A dynamic inflammatory cytokine network in the human ovarian cancer microenvironment. Cancer Res.

[6] Hussian S. P, Harris C.C. “Inflammation and cancer: an ancient link with novel potentials”. Int J Cancer 2007; 121(11): 2373–2380.10.1002/ijc.2317317893866

[7] Mills GB, May C, McGill M, Roifman CM, Mellors A (1988). A putative new growth factor in ascitic fluid from ovarian cancer patients: identification, characterization, and mechanism of action. Cancer Res.

[8] Freedman RS, Deavers M, Liu J, Wang E (2004). Peritoneal inflammation – a microenvironment for epithelial ovarian cancer (EOC). J Transl Med.

[9] Fang L, Xinjuan K, Qian D, Jin Y, Yuhu S (2014). Evaluation of tumor markers for the differerntial diagnosis of benign and malignant ascites. Ann Hepatol.

[10] Matte I, Lane D, Laplante C, Rancourt C, Piche A (2012). Profiling of cytokines in human epithelial ovarian cancer ascites. Am J Cancer Res.

[11] Lane D, Matte I, Rancourt C, Piche A (2011). Prognostic significance of IL-6 and IL-8 ascites levels in ovarian cancer patients. BMC Cancer.

[12] Lane D, Matte I, Garde-Granger P, Laplante C, Carignan A, Rancourt C (2015). Inflammation-regulating factors in ascites as predictive biomarkers of drug resistance and progression-free survival in serous epithelial ovarian cancers. BMC Cancer.

[13] Heng EC, Huang Y, Black SA, Trackman PC (2006). CCN2, connective tissue growth factor, stimulates collagen deposition by gingival fibroblasts via module 3 and alpha6- and beta1 integrins. J Cell Biochem.

[14] Chen N, Chen CC, Lau LF (2000). Adhesion of human skin fibroblasts to Cyr61 is mediated through integrin alpha 6 beta 1 and cell surface heparin sulfate proteoglycans. J Biol Chem.

[15] Grzeszkiewicz TM, Lindner V, Chen N, Lam SC, Lau LF (2002). The angiogenic factor cysteine-rich 61 (CYR61, CCN1) supports vascular smooth muscle cell adhesion and stimulates chemotaxis through integrin alpha (6) beta (1) and cell surface heparin sulfate proteoglycans. Endocrinology..

[16] Schober JM, Chen N, Grzeszkiewicz TM, Jovanovic I, Emeson EE, Ugarova TP, Ye RD, Lau LF, Lam SC (2002). Identification of integrin alpha (M) beta (2) as an adhesion receptor on peripheral blood monocytes for Cyr61 (CCN1) and connective tissue growth factor (CCN2): immediate-early gene products expressed in atherosclerotic lesions. Blood..

[17] Tsai MS, Bogart DF, Castaneda JM, Li P, Lupu R (2002). Cyr61 promotes breast tumorigenesis and cancer progression. Oncogene..

[18] Xie D, Yin D, Tong X, O’Kelly J, Mori A, Miller C (2004). Cyr61 is overexpressed in gliomas and involved in integrin-linked kinase-mediated Akt and β-catenon-TCF/Lef signaling pathways. Cancer Res.

[19] Zhou D, Herrick DJ, Rosenbloom J, Chaqour B (2005). Cyr61 mediates the expression of VEGF, αv-integrin, and α-actin genes through cytoskeletally based mechanotransduction mechanisms in bladder smooth muscle cell. J Appl Physiol.

[20] Lin J, Li N, Chen H, Liu C, Yang B, Ou Q (2015). Serum CYR61 is associated with clinical disease activity and inflammation in patients with systemic lupus erythematosus. Medicine (Baltimore).

[21] Choi JS, Kim KH, Lau LF (2015). The matricellular protein CCN1 promotes mucosal healing in murine colitis through IL-6. Mucosal Immunol.

[22] Lin J, Zhou Z, Huo R, Xiao L, Ooyang G, Wang L, Sun Y, Shen B, Li D, Li N (2012). Cyr61 induces IL-6 production by fibroblast-like synoviocytes promoting Th17 differentiation in rtheumatoid arthritis. J Immunol.

[23] Wu P, Ma G, Zhu X, Gu T, Zhang J, Sun Y, Xu H, Huo R, Wang B (2017). Cyr61/CCN1 is involved in the pathogenesis of psoriasis vulgaris via promoting IL-8 production by keratinocytes in a JNK/NF-kB pathway. Clin Immunol.

[24] Zhu X, Xiao L, Huo R, Zhang J, Lin J, Xie J, Sun S, He Y, Sun Y, Zhou Z, Shen B, Li N (2013). Cyr61 is involved in neutrophil infiltration in joints by inducing IL-8 production by fibroblast-like synoviocytes in rheumatoid arthritis. Arthritis Res Ther.

[25] Harris LG, Pannell LK, Singh S, Samant RS, Shevde LA (2012). Increased vascularity and spontaneous metastasis of breast cancer by hedgehog signaling mediated upregulation of Cyr61. Oncogene..

[26] D’Antonio KB, Toubaji A, Albadine R, Mondul AM, Platz EA, Netto GJ, Getzenberg RH (2010). Extracellular matrix associated protein CYR61 is linked to prostate cancer development. J Urol.

[27] Hou CH, Lin FL, Hou SM, Liu JF (2014). Cyr61 promotes epithelial-mesenchymal transition and tumor metastasis of osteosarcoma by Raf-1/MEK/ERK/Elk-1/TWIST-1 signaling pathway. Mol Cancer.

[28] Lo CW, Chen MW, Hsiao M, Wang S, Chen CA, Hsiao SM (2011). IL-6 trans-signaling in formation and progression of malignant ascites in ovarian cancer. Cancer Res.

[29] Nonna K, Kevin HE, Anm Nazmul HK, Kassondra SG, Kelly LS (2015). Cytokine profiling of ascites at primary surgery identifies an interaction of tumor necrosis factor-α and interleukin-6 in predicting reduced progression-free survival in epithelial ovarian cancer. Gynecol Oncol.

[30] Sun Y, Zhang J, Zhou Z, Wu P, Huo R, Wang B, Shen Z, Li H, Zhai T, Shen B, Chen X, Li N (2015). CCN1, a pro-inflammatory factor, aggravates psoriasis skin lesions bu promoting keratinocyte activation. J Invest Dermatol.

[31] Lin J, Huo R, Wang L, Zhou Z, Sun Y, Shen B, Wang R, Li N (2012). A novel anti-Cyr61 antibody inhibits breast cancer growth and metastasis in vivo. Cancer Immunol Immunother.

[32] Yang L, Cao X (2016). Characteristics and significance of pre-metastatic niche. Cancer Cell.

[33] Farajzadeh VS, Keshavarz-Fathi M, Silvestris N, Argentiero A, Rezaei N (2018). The role of inflammatory cytokines and tumor associated macrophages (TAMs) in microenvironment of pancreatic cancer. Cytokine Growth Factor Rev.

[34] Liao Z, Tan ZW, Zhu P, Tan NS. Cancer-associated fibroblasts in tumor microenvironment-Accomplices in tumor malignancy. Cell Immunol. 2018; Jan 31.10.1016/j.cellimm.2017.12.00329397066

[35] Yang L, Lin PC (2017). Mechanisms that drive inflammatory tumor microenvironment, tumor heterogeneity, and metastatic progression. Semin Cancer Biol.

[36] Voronov E, Apte RN (2017). Targeting the tumor microenvironment by intervention in interleukin-1 biology. Curr Pharm Des.

[37] Blank S, Nienhüser H, Dreikhausen L, Sisic L, Heger U, Ott K, Schmidt T (2017). Inflammatory cytokines are associated with response and prognosis in patients with esophageal cancer. Oncotarget..

[38] Ahmed N, Stenvers KL (2013). Getting to know ovarian cancer ascites: opportunities for targeted therapy-based translational research. Front Oncol.

[39] Reinart S, Schumann T, Finkernagel F, Wortmann A, Jansen JM, Meissner W (2014). Mixed-polarization phenotype of ascites-associated macrophages in human ovarian carcinoma: correlation of CD163 expression, cytokine levels and early relapse. Int J Cancer.

[40] Dijkgraaf EM, Heusinkveld M, Tummers B, Vogelpoel LT, Goedemans R, Jha V (2013). Chemotherapy alters monocyte differentiation to favour generation of cancer-supporting M2 macrophages in the tumor microenvironment. Cancer Res.

[41] Kotsopoulos J, Lubinski J, Gronwald J, Cybulski C, Demsky R, Neuhausen SL, Kim-Sing C, Tung N (2015). Factors influencing ovulation and the risk of ovarian cancer in BRCA1 and BRCA2 mutation carriers. Int J Cancer.

[42] Richards JS (2018). From follicular development and ovulation to ovarian cancers: an unexpected journey. Vitam Horm.

[43] Sapoznik S, Bahar-Shany K, Brand H, Pinto Y, Gabay O, Glick-Saar E, Dor C (2016). Activation-induced cytidine deaminase links ovulation-induced inflammation and serous carcinogenesis. Neoplasia..

[44] Cardenas C, Alvero AB, Yun BS, Mor G (2016). Redefining the origin and evolution of ovarian cancer: a hormonal connection. Endocr Relat Cancer.

[45] Benias PC, Wells RG, Sackey-Aboagye B, Klavan H, Reidy J, Buonocore D, Miranda M, Kornacki S, Wayne M, Carr-Locke DL, Theise ND (2018). Structure and distribution of an unrecognized interstitium in human tissues. Sci Rep.

[46] So KA, Min KJ, Hong JH, Lee JK (2015). Interleukin-6 expression by interactions between gynecologic cancer vells and human mesenchymal stem cells promotes epithelial-mesenchymal transition. Int J Oncol.

[47] Bachelot T, Ray-Coquard I, Menetrier-Caux C, Rastkha M, Duc A, Blay JY (2003). Prognostic value of serum levels of interleukin 6 and of serum and plasma levels of vascular endothelial growth factor in hormone-refractory metastatic breast cancer patients. Br J Cancer.

[48] Maccio A, Lai P, Santona MC, Pagliara L, Melis GB, Mantovani G (1998). High serum levels of soluble IL-2 receptor, cytokines, and C reactive protein correlate with impairment of T cell response in patients with advanced epithelial ovarian cancer. Gynecol Oncol.

[49] Gregory AD, Houghton AM (2011). Tumor-associated neutrophils: new targets for cancer therapy. Cancer Res.

